# Effect of Autoimmune Cell Therapy on Immune Cell Content in Patients with COPD: A Randomized Controlled Trial

**DOI:** 10.1155/2022/8361665

**Published:** 2022-01-10

**Authors:** Wen Li, Guanhong Li, Wei Zhou, Hui Wang, Yuqiong Zheng

**Affiliations:** Department of Respiratory and Critical Care Medicine, Chengdu First People's Hospital, Chengdu 610041, China

## Abstract

**Objective:**

To explore the effect of autoimmune cell therapy on immune cells in patients with chronic obstructive pulmonary disease (COPD) and to provide a reference for clinical treatment of COPD.

**Methods:**

Sixty patients with stable COPD were randomly divided into control group and treatment group (*n* = 30). The control group was given conventional treatment, and the treatment group was given one autoimmune cell therapy on the basis of conventional treatment. The serum levels of CD3+ T cells, CD4+ T cells, CD8+ cells, B cells, and NK cells in the peripheral blood were detected by flow cytometry. Possible adverse reactions were detected at any time during treatment.

**Results:**

There were no significant differences in the contents of CD3+ T cells, CD4+ T cells, CD8+ cells, B cells, and NK cells in the serum of the control group (*P* > 0.05). Compared with before treatment, the contents of CD3+ T cells, CD4+ T cells, CD8+ cells, B cells, and NK cells in the serum of the treatment group were significantly increased (*P* < 0.05). The ratio of CD4 + /CD8+ T cells in both control and treatment groups did not change significantly during treatment (*P* > 0.05). There were no significant differences in serum CD3+ T cells, CD4+ T cells, CD8+ cells, B cells, and NK cells in the treatment group at 30 days and 90 days after treatment (*P* > 0.05), but they were significantly higher than those in the control group (*P* < 0.05).

**Conclusion:**

Autoimmune cell therapy can significantly increase the level of immune cells in the body and can be maintained for a long period of time, which has certain clinical benefits for recurrent respiratory tract infections and acute exacerbation in patients with COPD.

## 1. Introduction

Chronic obstructive pulmonary disease (COPD) is a common chronic disease of respiratory system, with high morbidity, disability, and mortality [1]. COPD is the fourth leading cause of death in the world, and it is predicted that this disease will become one of the three leading causes of death in the population in 2021 [1, 2]. Exposure to environmental particles, especially cigarette smoke, is the most common cause of COPD. These patients exhibit a progressive airflow obstruction provoked by small airway fibrosis, alveolar wall destruction (emphysema), and chronic inflammation [3]. In the last decades, it has become evident that inflammatory cells play a key role in initiating and perpetuating the disease pathology.

COPD is a complex and progressive disease whose pathology is mainly driven and perpetuated by chronic inflammation. In fact, current treatments are mainly immunosuppressive drugs in combination with bronchodilators that mitigate the symptoms but do not cease disease progression. Inhaled corticosteroids (ICSs) are used extensively in the treatment of asthma and COPD due to their broad anti-inflammatory effects. They improve lung function, symptoms, and quality of life and reduce exacerbations in both conditions but do not alter the progression of disease. They decrease mortality in asthma but not COPD. Long-term treatment with ICSs is recommended by the GOLD guidelines for patients with an FEV1 < 50% predicted and/or frequent exacerbations and whose symptoms are not adequately controlled on long-acting bronchodilators, although long-term monotherapy with ICS is not recommended [4].

As the incidence rate of COPD increases, the deterioration of the disease brings a greater burden to the health care system, and more than 10 million of the annual visits outside the United States are planned. The direct cost of COPD treatment in the United States exceeds US $32 billion every year, which is estimated to account for 50% to 75% of these health care costs. Exacerbation is also an important outcome indicator of COPD [2].

In recent years, studies on COPD and immune function have attracted increasing attention. Immune function is the result of the interaction of various immune cells and cytokines, among which T lymphocytes, B lymphocytes, and NK cells are the important components of immune cells. Mature T cells can differentiate into different cell subsets such as CD3+CD4+CD8-T and CD3+CD4-CD8+ T cell subsets [3]. CD3+ is present on almost all T cells, and the total number of T cells can be calculated by measuring the number of CD3+ molecules. Activated CD4+ T cells release a variety of cytokines and coordinate the activity of other inflammatory cells. CD8+ T cells are a T cell subset that can kill infected or damaged cells but also cause the degradation and apoptosis of alveolar epithelial cells by releasing perforin, granzyme B, and tumor necrosis factor alpha (TNF-*α*) [4, 5]. When the ratio of CD4 + /CD8+ T cells is unbalanced, it generally indicates the immune dysfunction of the body. When COPD occurs, the levels of CD4+ T lymphocytes and CD4 + /CD8+ T lymphocytes in the peripheral blood serum of the body are significantly lower than those in healthy people [6]. The researchers found that the proportion of CD8+ T cells was strongly associated with COPD disease progression. During the exacerbation of COPD, CD4+ and CD8+ T cells in the peripheral blood of patients decreased [7, 8]. The above studies suggest that the levels of CD3+ T lymphocytes, CD4+ T lymphocytes, and CD4 + /CD8+ T lymphocytes in the peripheral blood of patients with COPD are positively correlated with COPD conditions, while the levels of CD8+ T lymphocytes are negatively correlated with COPD conditions.

Plasma cells, which are mainly differentiated from B lymphocytes, can secrete immune proteins and participate in the humoral immune process. Patients with COPD also have abnormal B lymphocyte count. Studies have shown that the number of B lymphocytes in the peripheral blood of COPD patients is significantly lower than that of the normal population. The density of CD3(+) and B cells in the small airway of patients with severe COPD was significantly higher than that in the parenchymal stroma. CD8+ cells increased in respiratory epithelial cells of patients with moderate COPD [9, 10]. These studies suggest that there is a deficiency of B lymphocytes in patients with COPD, and B lymphocytes may be involved in the process of immunopathological injury of COPD.

Natural killer (NK) cells, also known as natural immune cells, are mainly found in the peripheral blood and spleen and can play an anti-infection role by secreting inflammatory factors. NK cells can secrete cytokines after being activated in the immune process, inducing the generation of more NK cells to participate in the immune process together [11]. Studies have found that compared with healthy nonsmokers, the proportion of peripheral blood NK cells in COPD patients is lower [12]. Studies have shown that patients with COPD have immune dysfunction, and NK cells may be involved in the pathogenesis of COPD.

Autoimmune cells therapy (ACT) is a new therapeutic technique developed in recent years and a new direction of immunotherapy. ACT uses autoimmune cells, which not only can produce bidirectional regulation but also will not produce rejection reaction, and the immune function of patients can be improved in a short time. At present, ACT is mainly used in tumors and diseases of the hematological system [13–15], while there are few reports on other diseases, such as COPD. Therefore, this study expanded the observation sample size, selected severe COPD as the research object, and explored the influence of ACT treatment on the peripheral blood immune cell content of COPD patients, aiming at providing new clinical evidence for the use of ACT in the treatment of COPD.

## 2. Objects and Methods

### 2.1. Subjects

#### 2.1.1. Case Selection

All patients were enrolled according to the diagnostic criteria of COPD [16]. The inclusion and exclusion criteria and abort test standard are listed in Table 1.

#### 2.1.2. Test Scheme

A total of 60 patients with stable COPD in group D were included in this study. The subjects were all outpatients who visited Chengdu First People's Hospital from January 2016 to December 2018. According to the order of treatment, they were divided into two groups (*n* = 30). The treatment group was treated with traditional therapy in combination of autoimmune cell therapy for once.

### 2.2. Treatment Options

Sixty COPD patients in stable phase D group were selected and divided into control group and treatment group (*n* = 30) (Figure 1, Table 2). The control group was given conventional oxygen inhalation, bronchodilator, phlegm-reducing drugs, and anti-inflammatory treatment, while the treatment group was given one autoimmune cell therapy on the basis of conventional treatment (Figure 2).

### 2.3. Collection and Treatment of Autoimmune Cells

#### 2.3.1. Evaluation and Preparation

Patients needed to review the relevant examination report and be informed of precautions before collection (Table 3).

#### 2.3.2. Cell Collection

A disposable 50 ml syringe, a disposable No. 7 or No. 12 venous blood sampling needle, a sterile cloth, and an anticoagulant (heparin sodium (12500 U/2 ml)) were prepared. The test report and informed consent were checked. Patient's information and treatment plan were also checked. After all were correct, the mark was filled on the syringe. Labels with patient information should be affixed to the syringe and be careful not to cover the scale. Lay aseptic treatment was tried for collection of blood samples. Patients' information was checked before blood collection. Large and thick vessels in the elbow were routinely selected, such as the basilic vein, median vein, or cephalic vein (to avoid scar and skin lesions). The aseptic technique was performed strictly, and the puncture was performed according to the conventional superficial venipuncture technique.

#### 2.3.3. Postacquisition Processing

After the collection was completed, the blood needle was pulled out immediately, and the puncture site was pressed for 5-10 minutes. After the puncture site was checked for no bleeding, the patient was sent back to the ward, ordered to rest in bed for 30-60 minutes, and given warm boiled water orally as appropriate. The blood was drawn from the blood collection needle into the syringe, put back into the needle sleeve, tightened, tied the tube, and fixed. After rechecking the marking information on the syringe, the blood sample was put in a sterile cloth and wrapped; it was put into the delivery box and sealed. The delivery personnel were asked to be sent to the laboratory for separation and culture. Copies of the immunocell therapy sheet and relevant test reports were sent back to the laboratory with the blood sample for archiving.

#### 2.3.4. Laboratory Treatment

50 ml of peripheral venous blood was extracted, and heparin sodium was used as anticoagulant. Mononuclear cells were isolated with the Ficoll solution (2000 rpm, 20 min) and washed twice with normal saline (1600 rpm, 5 min) by the density gradient centrifugation method. Then mononuclear cells were transferred to the T75 culture flask. 30 ml DC-CIK cell special medium containing 5%~10% autologous plasma was added into culture flask. The culture was placed in an incubator at 37°C and 5% CO2. Cell morphology and proliferation were observed every day, timely hydration or passage. After being cultured for about 7 days, all cells were collected in a centrifuge tube, and the supernatant was centrifuged (1600 rpm, 5 min) and then washed twice with normal saline (1600 rpm, 5 min). A small number of cells were taken for counting, and cell or survival rate was observed. The cells were resuspended in a 100 ml saline injection and returned to the patient within 4 h.

### 2.4. Peripheral Blood Cell Test

#### 2.4.1. Whole Blood Treatment

4 ml peripheral blood of sodium citrate was collected for anticoagulation. Mononuclear cells were isolated from whole blood with lymphatic separation solution (Ficoll). After mixing the blood : PBS = 1 : 1, a centrifuge tube was prepared with Ficoll to 15 ml at room temperature according to the mixture of blood : Ficoll = 1 : 1. The mixture was slowly added to the Ficoll surface, rising slowly and descending quickly (400 g, 20 min). The white cloud film was carefully precipitated to a clean 15 ml centrifuge tube. 5 ml PBS was added into it and was washed at 2000 rpm for 5 min. Then the supernatant was discarded and repeated for one time.

#### 2.4.2. Staining and Testing

50 *μ*l cells were precipitated into the flow tube, cell membrane antibodies CD4+, CD8+, B cells, and NK cells were successively added with 5 *μ*l each, and the mixture was mixed at 4°C for 30 min. The mixture was washed with 2 ml PBS (2000 rpm, 5 min), and the supernatant was discarded. 50 *μ*l of kit solution 1 was added and mixed well at room temperature for 15 min. The mixture was washed with 2 ml PBS (2000 rpm, 5 min), the supernatant was discarded. 50 *μ*l of the kit solution 2 was added and mixed well at room temperature for 5 min. 5 *μ*l of individual intracellular antibodies (Table 4) CD4+/CD8+/B cells/NK cells was added and mixed at room temperature for 30 min. The mixture was washed with 2 ml PBS, centrifuged at 2000 rpm for 7 min, and repeated for one time. The sample was examined by flow cytometry.

### 2.5. Observation Indicators

Basic biological indicators of COPD patients were recorded, including sex, age, height, weight, disease duration, smoking status, complications, temperature, pulse, respiration, and blood pressure. The changes of T cell subsets, B cells, and NK cell contents in the peripheral blood of patients with COPD were detected. Adverse reactions occurred during the test were recorded, mainly including blood routine, creatinine, urea nitrogen, transaminase, bilirubin, and electrocardiogram.

### 2.6. Statistical Analysis

All data were analyzed by using the IBM SPSS Statistics 21.0 software package. The data were represented as mean ± standard deviation (SD), in line with normal distribution and homogeneity of variance, and *t* test was used. Unnormal distribution or variance was analyzed by the rank sum test. Enumerative data were described by frequency and analyzed by Pearson's chi-square test. *P* < 0.05 indicated that the difference was statistically significant.

### 2.7. Medical Ethics

Strictly following the declaration of Helsinki, this study was carried out in accordance with the strict specification of China medical research, which had passed the Chengdu First People's Hospital Medical Ethics Committee approval. Prior to enrollment, all patients would be fully briefed by writing to them or their designated family members on the purpose, procedures, and possible risks of the clinical study, and patients would be informed of their right to withdraw at any time. All patients in this study were provided with a written patient informed consent before entering the study, and only after obtaining informed consent of each subject could patients be enrolled in the study.

## 3. Results

### 3.1. Basic Information

A total of 60 patients with COPD who were in line with group D were included in this study, all of whom were admitted to Chengdu First People's Hospital from January 2016 to December 2018. They were divided into two groups according to the order of treatment and the patients' wishes. There was no loss during follow-up in the control group, while 1 patient with acute exacerbation within 3 months after the start of the study was excluded from the treatment group. There were 30 patients in the control group and 29 patients in the treatment group who completed the study. There was no significant difference between the two groups in gender, age, height, weight, BMI, smoking history, diabetes mellitus, hypertension, and course of disease (*P* > 0.05), and the baseline was comparable (Table 5).

### 3.2. Changes of Serum T Cell Subsets in Two Groups of COPD Patients

#### 3.2.1. Serum CD3+ T Cell Content in COPD Patients

The serum CD3+ cell content in the peripheral blood of the treatment group at 30 days and 90 days after treatment was significantly higher than that before treatment. At 30 days and 90 days after treatment, there were statistical differences between the treatment group and the control group, and the treatment group was significantly higher than the control group (Table 6, Figure 3).

#### 3.2.2. Serum CD4+ T Cell Content in COPD Patients

In the treatment group, the serum CD4+ T cell content increased significantly after 30 days and 90 days of treatment. There was no statistical difference in serum CD4+ T cell content between the treatment group at 30 and 90 days after treatment. On day 30 and 90 after treatment, the serum CD4+ T cell content of the treatment group was higher than that of the control group (Table 7, Figure 4).

#### 3.2.3. Serum CD8+ T Cell Content in COPD Patients

In the treatment group, the serum CD8+ T cell content increased significantly 30 and 90 days after treatment. There was no significant difference in serum CD8+ T cell content between the treatment group at 30 days and 90 days after treatment. On day 30 and day 90, the serum CD8+ T cell content of the treatment group was significantly higher than that of the control group (Table 8, Figure 5).

#### 3.2.4. The Ratio of CD4 + /CD8+ T Cell in COPD Patients

Before and after treatment, there was no statistical difference in the ratio of CD4 + /CD8+ T cells between the control group and the treatment group (Table 9, Figure 6).

### 3.3. Serum B Cell Content of COPD Patients

Compared with before treatment, the serum B cell content of the treatment group increased on the 30th and the 90th days after treatment, and there was no statistical difference in the B cell level after treatment for the 30th and the 90th days, suggesting that the efficacy of ACT treatment was sustainable. At 30 and 90 days after treatment, B cell levels in the treatment group were significantly higher than those in the control group (Table 10, Figure 7).

### 3.4. Serum NK Cell Content in COPD Patients

The serum level of NK cells in the treatment group was significantly higher than that before treatment at 30 and 90 days after treatment. There was no significant difference in the level of NK cells in the treatment group at 30 days and 90 days after treatment. On days 30 and 90 after treatment, the level of NK cells in the treatment group was significantly higher than that in the control group (Table 11, Figure 8).

## 4. Discussion

COPD is a chronic and incomplete reversible respiratory disease with airflow restriction as the main clinical feature [16]. Patients with COPD may intermittently experience acute exacerbation of respiratory symptoms, which is called acute exacerbation. And the rate of disability and mortality in patients with acute exacerbation increases significantly [17]. For patients with COPD, several causes of exacerbation are recommended, such as heart failure, pneumonia, pulmonary embolism, and noncompliance with inhaled drugs or inhaled irritants, such as tobacco smoke or particles. The most common cause is viral or bacterial infection. Among the patients hospitalized for acute exacerbation of COPD, viral infection, bacterial infection, or both were detected in 78% of cases. More importantly, the acute exacerbation was more serious than that of patients with noninfectious causes, showing more obvious damage to lung function and longer hospitalization time [1–3].

Epidemiological studies have found that COPD is closely related to genetic and environmental factors, and the incidence of COPD in susceptible populations is generally familial. External factors (such as respiratory tract infection) and internal factors (airway hyperresponsiveness, etc.) are also involved in the pathogenesis of COPD [18]. Poor lifestyle preferences can contribute to the risk of COPD infection, and smoking is a common risk factor. Nicotine and other components in cigarettes can damage lung tissue, which may lead to pulmonary fibrosis, thereby affecting lung function, and significantly increasing the prevalence of COPD [19–21].

Among COPD patients, there is a high demand for safe and effective anti-inflammatory treatments, which can not only prevent the deterioration of the disease but also have a beneficial effect on the course of the disease and improve survival. Although there are several new methods designed to target chronic neutrophilic lung inflammation itself in COPD patients, strategies to target the underlying causes of lung neutrophilic inflammation may be better for success. In two chronic airway diseases (especially in more difficult and complex situations), the choice of the best treatment should be based not only on arbitrary clinical markers but also on the underlying immunopathology.

Increased neutrophils and macrophages in the lungs can quickly identify inflammation. In fact, inflammation caused by macrophages is one of the main causes of abnormal immune responses. It is believed that most of these macrophages are derived from bone marrow-derived blood mononuclear cells, which are quickly recruited to the injury site rather than the expansion of macrophages in the lung tissue. Studies have shown that decreased or disorder of immune function plays a key role in the occurrence and development of COPD, mainly with decreased cellular immune function [22]. Patients with COPD usually have abnormal immune T cells. Syrjälä et al. [23] analyzed the immune factors. The results showed that the ratio of CD4 + /CD8+ was an important indicator of disease change in the body, and the ratio of CD4 + /CD8+ would decrease after repeated infection and exacerbation of disease. The imbalance of T cell subsets in patients with COPD leads to a decline in immune function and further aggravation of the disease. After immunoanalysis of CD4+ and CD25+ in patients with COPD, researchers found that T lymphocyte levels were significantly lower, and after antibiotic treatment, the level of immune cells increased, but still lower than normal [24].

Abnormal immune function of COPD affects the development and prognosis of COPD. As a means of regulating immune function, autoimmune cell therapy may have a potential unique advantage in the treatment of COPD. The autoimmune cells used in this study were especially cultured in a laminar flow laboratory in accordance with the national GMP standard, and a group of enhanced dendritic cells (DC), cytokine-induced killer (CIK) cells, NK cells, T cells, NKT cells, CTL cells, and other immune cells was obtained and then transplanted into the patients. DC is one of the professional antigen presenting cells, whose main function is the uptake, processing, processing, and presentation of antigen. Myeloid DC is mainly involved in stimulating the immune response of T cells, while lymphoid DC is involved in antiviral innate immunity by secreting high levels of type I interferon [25]. CIK, (cytokine-induced killer) cells are a kind of heterogeneous cell population induced by Schmidt-Wolf from peripheral blood monocytes in the mid-1980s, expressing both CD3 and CD56 membrane protein molecules. CIK possesses both the strong tumoricidal activity of T lymphocytes and the non-MHC restriction of NK cells. Therefore, they are also known as NK cell-like T lymphocytes, which have functions such as enhancing immunity, antitumor, and anti-infection [26]. DC and CIK are mutually beneficial and complementary in the immune system of the body. Compared with homologous cells, the double-clonal immune cells produced under coculture have more powerful properties of killing tumor cells, improving immunity, and inhibiting tumor growth [27]. DC-CIK immunotherapy has been widely used in the clinical treatment of malignant tumors with remarkable effects, but there is no relevant report on the treatment of COPD.

In this study, patients in the treatment group were given 1 time of autoimmune cell therapy on the basis of conventional treatment to achieve two-way regulation of immune function in COPD patients. After 2 years of study, it was found that autoimmune cell therapy for COPD affected the changes of immune cell levels in the body. T cells are an important type of immune cells that interact with each other to maintain the normal operation of the immune system. The disorder of T cell subsets is the main cause of immune disorders in COPD [28, 29]. When the ratio of CD3 + , CD4 + , CD4+/CD8+ T decreases or the level of CD8+ T increases, it indicates that the immune function of the body is weakened. In this study, CD3+ T, CD4+ T, and CD8+ T levels were not significantly changed in the control group, while serums CD3+ T and CD4+ T were increased to a certain extent in the treatment group after 30 and 90 days of treatment with autoimmune cells. It is suggested that ACT may regulate the cellular immunity level of COPD patients by upregulating the levels of CD3+, CD4+, and CD8+ T cells in patients with stable COPD. This is consistent with the results of previous studies, suggesting that autoimmune cell therapy can increase the levels of CD3+ T and CD4+ T lymphocytes in COPD patients and improve the cellular immune function of the body.

Some studies have suggested that the increase of CD8+ T cells is a negative factor for COPD patients, and even in some studies, it has been suggested that the application of small dose of azithromycin can reduce the number of CD8+ T cells in the alveolar lavage fluid of COPD patients, reduce the level of granulosin B released by CD8+ T cells in the peripheral blood, and improve the cellular immunity of COPD patients [30]. In this study, CD8+ T level was upregulated after autoimmune cell therapy, which has not been seen in other previous studies on the treatment of COPD, and the literature on autoimmune cell therapy of COPD is limited, so the reasons for the increase of CD8+ T level and the advantages and advantages of the increase of CD8+ T level on COPD still need to be further studied. This study also showed that there was no statistical difference in CD4 + /CD8+ T ratio, possibly because the autoimmune cell therapy had the same regulation on the T cell subgroup of patients, all of which were ascending regulation.

Studies have shown that B lymphocytes have a low level of both BAFL and serum in COPD patients [31], indicating a low level of humoral immunity in COPD patients. Decrease of humoral immunity can lead to increased risk of airway infection, which is directly related to acute exacerbations in patients. There is excessive humoral immunity in some patients with COPD, and hormone therapy can reduce the adaptive immunity in patients with COPD and can effectively treat patients with enhanced B cell/antibody response [32]. The results of this trial showed no significant change in B lymphocyte levels in stable COPD patients receiving conventional treatment for 90 days, whereas B lymphocyte levels were significantly increased in patients receiving autoimmune cell therapy at 30 days and 90 days. It is suggested that autoimmune cells can upregulate the humoral immunity level of COPD patients, which is consistent with the above research results. It suggests that ACT treatment can improve humoral immune function in COPD patients.

NK cells sense viral infection, transformed or stressed cells in an antigen-nonspecific way, and then secretes a series of cytokines, such as IFN-*γ*, TNF-*α*, and IL-12, which play a role in destroying viral infection and transformed cells. Studies have found that exposure of human NK cells to cigarette smoke can inhibit the production of IFN-*γ* and TNF-*α* and the expression of perforin [33]. Although the number and function of NK cells in the lungs of healthy smokers and COPD smokers are controversial, reduced NK cell activity has been observed in the blood of patients with COPD [34]. Besides, in the context of disease, macrophages can acquire different phenotypes to meet the needs of the local microenvironment. It is generally believed that there are two main phenotypes: activated (M1) and replacement (M2) macrophages, which were originally defined according to the in vitro settings. M1 responds to type 1 driven inflammation by secreting IL-12a or TNF-*α* and other inflammatory cytokines, while M2 is induced by type 2 stimulation and participates in tissue remodeling, anti-inflammatory response, and cellular effects. During COPD, changes in lung biology and the pleiotropic effect and plasticity of macrophages result in continuous phenotypic changes, making it difficult to distinguish between M1 and M2. In fact, it has been assumed that there are at least 8 different phenotypes [35].

In this study, the NK cells of COPD patients in the control group were at a low level and showed no significant change within 3 months. However, the NK cells gradually increased after ACT treatment and were still at a high level after 30 days and 90 days of treatment. In conclusion, ACT treatment can improve serum NK cell level and immune level in patients with COPD, thus enhancing the anti-inflammatory and antiviral ability of the body.

## 5. Conclusion

To sum up, this study analyzed the dynamic changes of relevant immune cells during the pathogenesis by exploring the changes of immune cell levels in patients with COPD under different treatment modes, which strengthened the cognition of clinical treatment methods of COPD and provided a theoretical basis for clinical treatment of COPD. The proportion of cells in vivo was still higher than that of patients in the conventional treatment group, suggesting that autoimmune cell therapy can not only improve the immune level of patients but also last for a long time, which has clinical benefits for patients with recurrent respiratory tract infections and acute exacerbations.

## Figures and Tables

**Figure 1:** The grouping scheme for COPD patients. Note: the grading standard was that FEV1 accounted for % of the expected value. Level 1: mild; level 2: moderate; level 3: severe; level 4: extremely severe.

**Figure 2:** The flow chart of the test.

**Figure 3:** Proportion of CD3+ cells in the peripheral blood serum (%). The serum of CD3+ cell content in the peripheral blood of the treatment group at 30 days and 90 days after treatment was determined. Note: ^∗^*P* < 0.05 vs. the control group; ∗∗*P* < 0.01 vs. the control group; ^△^*P* < 0.05 vs. in the same group before treatment.

**Figure 4:** Proportion of CD4+ cells in the peripheral blood serum (%). The serum of CD4+ cell content in the peripheral blood of the treatment group at 30 days and 90 days after treatment was determined. Note: ^∗^*P* < 0.05 vs. the control group; ^△^*P* < 0.05 vs. in the same group before treatment.

**Figure 5:** Proportion of CD8+ cells in the peripheral blood serum (%). The serum of CD8+ cell content in the peripheral blood of the treatment group at 30 days and 90 days after treatment was determined. Note: ^∗^*P* < 0.05 vs. the control group; ^△^*P* < 0.05 vs. in the same group before treatment.

**Figure 6:** Serum CD4 + /CD8+ T cell ratio in the peripheral blood serum (%). The serum of CD4 + /CD8+ cell content in the peripheral blood of the treatment group at 30 days and 90 days after treatment was determined.

**Figure 7:** Proportion of B cells in the peripheral blood serum (%). The serum of B cell content in the peripheral blood of the treatment group at 30 days and 90 days after treatment was determined. Note: ^∗^*P* < 0.05 vs. the control group; ^△^*P* < 0.05 vs. in the same group before treatment.

**Figure 8:** Proportion of NK cells in the peripheral blood serum (%). The serum of NK cell content in the peripheral blood of the treatment group at 30 days and 90 days after treatment was determined. Note: ^∗^*P* < 0.05 vs. the control group; ^△^*P* < 0.05 vs. in the same group before treatment.

**Table 1:** Inclusion and exclusion criteria and abort test standard.

Project	
Inclusion criteria	FEV1/FVC < 0.70 after inhalation of bronchodilators, except for other diseases causing incomplete reversible airflow obstruction
	45-80 years old
	Patients without other major diseases, history of allergies, and genetic history
	Signed informed consent

Exclusion criteria	Patients with chronic cough and wheezing caused by tuberculosis, tumor, irritant gas allergy etc.
	Patients complicated with cardiovascular, liver, kidney, hematopoietic system, and other serious primary diseases
	Patients with abnormal behavior or mental illness
	Allergic people
	Patients with communication barriers
	Patients with acute aggravation within 3 months of treatment
	Suffer from other major diseases and were allergic to the drugs used in this study
	Patients without using the drug as prescribed
	Those whose efficacy or safety judgment was affected by incomplete data

Abort test standard	Patients with severe adverse reactions or special physiological changes
	Patients with life-threatening

**Table 2:** Grouping scheme of COPD patients.

Classification	Characteristics		Lung function classification	Acute exacerbation/year	mMRC	CAT
	Risk level	Symptoms				
A	Low	Less	GOLD 1-2	≤1	0-1	<10
B	Low	More	GOLD 1-2	≤1	≥2	≥10
C	High	Less	GOLD 3-4	≥2	0-1	<10
D	High	More	GOLD 3-4	≥2	≥2	≥10

**Table 3:** Preparation matters before cell collection.

Project	Indicators
Number of peripheral white blood cells	≥6 × 10^9^/l
Psychology of patients	1. Explain the purpose of treatment and the basic operating procedures to the patients and their families 2. Increase its predictability, reduce ideological concerns, and sign the informed consent
Essential inspection item	Blood routine, 8 infectious diseases (5 hepatitis B, syphilis, HIV/AIDS, and hepatitis C)
Blood vessels to prepare	Choose large, thick, straight, unsuitable for sliding, and good elasticity vessels to avoid needle insertion in phlebitis, abrasion, sclerosis, scar, and skin damage
Work and rest	Get enough sleep to avoid catching cold
Dietary guidelines	1. One day before collection, a light diet rich in iron and calcium should be eaten, and greasy food should be abstained
	2. Fasting was required on the day of cell collection
	3. 10~20 ml 10% calcium gluconate injection was taken orally 20 min before collection to prevent citrate reaction

**Table 4:** Antibodies used for flow cytometry.

Antigen	Fluorochrome	Isotype	Clone	Source
CD4	FITC	Mouse IgG1	OKT4	Beckman Coulter, Luton, UK
CD8a	APC eFluor 780	Mouse IgG1	RPA-T8	Beckman Coulter, Luton, UK
B cells	FITC eFluor650	Mouse IgG1	CHY5	Beckman Coulter, Luton, UK
NK cells	FITC eFluor723	Mouse IgG1	HSP-YK	Beckman Coulter, Luton, UK
CD3	FITC eFluor590	Mouse IgG1	SJK-7	Beckman Coulter, Luton, UK

**Table 5:** Basic information of COPD patients in the two groups.

Project	Control group (*n* = 30)	Treatment group (*n* = 29)	*χ* ^2^/*t*	*P*
Gender (M/F)	19/11	15/14	0.814	0.367
Age (years)	71.93 ± 5.24	70.79 ± 6.23	1.990	0.164
Height (cm)	161.80 ± 5.69	162.3 ± 7.49	1.415	0.239
Weight (kg)	62.06 ± 5.05	61.13 ± 8.46	1.127	0.138
BMI (kg/m^2^)	23.74 ± 1.97	23.18 ± 2.89	2.685	0.107
Smoking history (*n*)	12	13	0.141	0.798
Complicated diabetes mellitus (*n*)	6	3	1.063	0.302
Complicated with hypertension (*n*)	8	10	0.425	0.514
Course of disease (year)	10.25 ± 2.13	11.04 ± 2.45	1.125	0.139

**Table 6:** Proportion of CD3+ cells in the peripheral blood serum of each group (%).

Project	Control group (*n* = 30)	Treatment group (*n* = 29)	*t*	*P*
Before treatment	63.15 ± 17.70	64.94 ± 10.94	0.727	0.470
30 days after treatment	63.73 ± 11.71	72.86 ± 15.26^∗∗^^△^	4.125	≤0.001
90 days after treatment	63.01 ± 12.92	71.81 ± 8.69^∗∗^^△^	4.555	≤0.001

Note: ^∗^*P* < 0.05 vs. the control group; ^∗∗^*P* < 0.01 vs. the control group; ^△^*P* < 0.05 vs. in the same group before treatment.

**Table 7:** Contents of CD4+ cells in the peripheral blood serum of each group (%).

Project	Control group (*n* = 30)	Treatment group (*n* = 29)	*t*	*P*
Before treatment	30.47 ± 7.67	30.65 ± 9.51	0.081	0.936
30 days after treatment	29.38 ± 6.13	36.50 ± 6.76^∗^^△^	4.240	0.002
90 days after treatment	29.47 ± 4.70	35.56 ± 5.69^∗^^△^	4.478	0.001

**Table 8:** Contents of CD8+ cells in the peripheral blood serum of each group (%).

Project	Control group (*n* = 30)	Treatment group (*n* = 29)	*t*	*P*
Before treatment	24.39 ± 7.21	25.65 ± 9.45	0.580	0.564
30 days after treatment	24.04 ± 6.46	28.72 ± 8.06^∗^^△^	2.462	0.017
90 days after treatment	24.23 ± 5.57	28.65 ± 5.71^∗^^△^	3.007	0.004

**Table 9:** Serum CD4 + /CD8+ T cell ratio in each group.

Project	Control group (*n* = 30)	Treatment group (*n* = 29)	*t*	*P*
Before treatment	1.40 ± 0.63	1.32 ± 0.50	0.530	0.599
30 days after treatment	1.33 ± 0.51	1.35 ± 0.37	0.101	0.920
90 days after treatment	1.30 ± 0.44	1.27 ± 0.26	0.312	0.756

**Table 10:** Comparison of proportion of B cells in the peripheral blood serum between two groups (%).

Project	Control group (*n* = 30)	Treatment group (*n* = 29)	*t*	*P*
Before treatment	8.59 ± 5.08	8.26 ± 4.69	0.256	0.799
30 days after treatment	8.62 ± 4.55	11.99 ± 4.47^∗^^△^	2.863	0.006
90 days after treatment	9.54 ± 4.47	11.95 ± 3.54^∗^^△^	2.289	0.026

**Table 11:** Comparison of proportion of NK cells in the peripheral blood serum between two groups (%).

Project	Control group (*n* = 30)	Treatment group (*n* = 29)	*t*	*P*
Before treatment	8.73 ± 4.19	8.81 ± 4.22	0.068	0.946
30 days after treatment	9.04 ± 3.86	11.84 ± 4.00^∗^△	2.767	0.009
90 days after treatment	8.86 ± 3.06	12.65 ± 4.69∗∗△	4.297	≤0.001

## Data Availability

The authors confirm that the data supporting the findings of this study are available within the article.
